# In Silico Identification of Hub Genes as Observing Biomarkers for Gastric Cancer Metastasis

**DOI:** 10.1155/2022/6316158

**Published:** 2022-04-30

**Authors:** Arulprakasam Ajucarmelprecilla, Jhansi Pandi, Ranjithkumar Dhandapani, Saikishore Ramanathan, Jayaprakash Chinnappan, Ragul Paramasivam, Sathiamoorthi Thangavelu, Abdul-Kareem Mohammed Ghilan, Saad Ali S. Aljohani, Atif Abdulwahab A. Oyouni, Abdullah Farasani, Malik A. Altayar, Hussam Awwadh E. Althagafi, Othman R. Alzahrani, Kaliannan Durairaj, Anupama Shrestha

**Affiliations:** ^1^Medical Microbiology Unit, Department of Microbiology, Alagappa University, Karaikudi, Tamil Nadu, India; ^2^Chimertech Private Limited, Chennai, India; ^3^Department of Bioinformatics, Bharathiar University, Coimbatore, Tamil Nadu, India; ^4^Department of Botany and Microbiology, College of Science, King Saud University, P.O. Box 2455, Riyadh 11451, Saudi Arabia; ^5^Department of Basic Medical Sciences, Faculty of Medicine, Alrayan Colleges, Almadinah Almunawarah, Saudi Arabia; ^6^Department of Biology, Faculty of Sciences, University of Tabuk, Tabuk, Saudi Arabia; ^7^Genome and Biotechnology Unit, Faculty of Sciences, University of Tabuk, Tabuk, Saudi Arabia; ^8^Biomedical Research Unit, Medical Research Center, Jazan University, Jazan 45142, Saudi Arabia; ^9^Department of Medical Laboratory Technology, College of Applied Medical Sciences, Jazan University, Jazan 45142, Saudi Arabia; ^10^Department of Medical Laboratory Technology, Faculty of Applied Medical Sciences, University of Tabuk, Tabuk, Saudi Arabia; ^11^Biology Department, Faculty of Science and Arts, Al-Mikhwah, Al-Baha University, Saudi Arabia; ^12^Zoonosis Research Center, School of Medicine, Wonkwang University, Iksan, Republic of Korea; ^13^Research Institute of Agriculture and Applied Science, Tokha Kathmandu 2356, Nepal; ^14^Department of Plant Protection, Himalayan College of Agricultural Sciences and Technology, Kalanki, 44600 Kathmandu, Nepal

## Abstract

Perception of hub genes engaged in metastatic gastric cancer (mGC) promotes novel ways to diagnose and treat the illness. The goal of this investigation is to recognize the hub genes and reveal its molecular mechanism. In order to explore the potential facts for gastric cancer, the expression profiles of two different datasets were used (GSE161533 and GSE54129). The genes were confirmed to be part of the PPI network for gastric cancer pathogenesis and prognosis. In Cytoscape, the CytoHubba module was used to discover the hub genes. Responsible hub genes were identified. Data from Kaplan–Meier plotter confirmed the predictive value of these distinct genes in various stages of gastric malignancy. Upregulated and downregulated genes were identified to utilize for further analysis. Positive regulation by a host of viral process, positive regulation of granulocyte differentiation, negative regulation of histone H_3_–K_9_ methylation were found in DEGs analysis. In addition, five KEGG pathways were identified as an essential enhancer that include nucleotide excision repair; base excision repair; DNA replication; homologous recombination; and complement and coagulation cascades. POLE, BUB1B, POLD4, C3, BLM, CCT7, PRPF31, APEX1, PSMA7, and CDC45 were chosen as hub genes after combining the PPI results. Our study recommends that BUB1B, CCT7, APEX1, PSMA7, and CDC45 might be potential biomarkers for gastric cancer. These biomarkers are upregulated genes. Therefore, suppression of these genes will increase the survival rate in gastric cancer patients.

## 1. Introduction

Gastric threatening is the most notable complication behind this infection worldwide. Gastric cancer mortality is leading with 784,000 cases around the worldwide [1]. Genetic factor and food sources are the main peril in gastric cancer development [2]. Most gastric cancer conflicts exist from familial aggregation (more than 10%). General threats of gastric cancer are weight loss, dyspepsia, stomach torture, and anorexia. In addition, sickliness might be accessible in depleting malignancies. Earlier gastric patient's progressive operations are higher than postoperative; past five years perseverance rate is 90%, and early gastric threats are commendable based on therapeutic effects. According to the findings, quality verbalizations in cells are controlled at both the transcriptional and post-transcriptional phases. Record factors (TFs) organize quality records, similar to mRNA corruption and protein understanding, whilst miRNAs oversee quality verbalization by interfering with post-transcriptional activities [3]. In the complex scenario of expressing DNA plans, proteins act as record factors to control the rate at which innate information is transferred from DNA to mRNA [4]. miRNAs are short noncoding RNAs found in cells that have a function in RNA silence and the explanation of post-transcriptional value [5]. In a subset of patients with defused gastric infections, hereditary gastric hazardous development (HDGC) problem is linked to heterogeneous germline changes in E-cadherin (E-cad) in any case termed CDH1 quality in a group of people with defused gastric infections; recurrence of HDGC attributable to germline CDH1 modification ranges from 1% to 3% [6]. CDH1 encoded the tumor silencer protein E-cadherin, as the hereditary reason behind acquired GC (HDGC); CDH1 mutation increases the lifetime hazard of diffuse gastric cancer (DGC) and lobular chest ailment.

Microarrays are normally used to separate DNA, mRNA, proteins, and other natural combinations [6]. Microarray assessment is used in quality verbalization profiling where a tremendous proportion of information is ordinarily made. It is essential to outfit the natural comprehension with real significance. Even with biomarkers and restorative targets found in gastric cancer, it is critical for expanding the determination. In spite of these reasons, treatment of gastric cancer remains not successful [29]. Gene expression omnibus (GEO) datasets ([7] and Cancer Genome Atlas Research N, 2014) were widely used to uncover promising biomarkers for malignancy detection, new therapy targets and visualization expectation as of late, and has given a valuable method to clarify basic genome modification in carcinogenesis. Besides, addressing irregularities in research results are tough because of the utilization of various microarray stages or restricted sample size. Coordinating bioinformatics approaches have got more often embraced in malignancy research and progression; these results have been documented [8]. We found DEGs between TT vs. NT in gastric tumor datasets. This study illuminates the idea of identifying the probable therapeutic biomarkers that were linked with gastric malignancy (Figure 1). In this work, a gene expression profile with accession number GSE161533 and GSE54129 were selected from the GEO, in which, Gene Expression Omnibus informational index provides much information about microarray experiment datasets. GEO2R was used to determine DEGs and further bioinformatic analyses such as biological processes, molecular functions, and cellular components in Gene Ontology and pathway enrichment were done. PPI network was built for recognizing the center qualities from the outcome. The above study might contribute in understanding the mechanism of potential biomarkers identified for gastric carcinoma metastasis.

## 2. Materials and Methods

### 2.1. Microarray Data Sources

The Gene Expression Omnibus database yielded 11386 datasets of human gastric carcinoma for the phrase given as ‘gastric malignancy.' From this search, two datasets (GSE161533 and GSE54129) were selected and used for this work. The Agilent GPL570 stage ([HG-U133_Plus_2] Affymetrix Human Genome U133 plus 2.0 Array) was utilized by GSE54129. The GSE161533 dataset was reliant onstage ([HG-U133_Plus] Affymetrix Human Genome U133 plus 2.0 Array). DEGs were acquired by the measures of logFC (fold change) in upregulated ≥1.5 and downregulated genes ≤ minus 1.5, adjusted *p* value < 0.05. GSE161533 and GSE54129 were chosen for consecutive study along with the following criteria: DEGs between gastric malignancy tissues vs. normal surrounding tissue were investigated using the *R* language in Limma package.

### 2.2. Analysis of GO and Enrichment

Gene ontology clarifies the function of differentially expressed genes. Enrichr, a free online enrichment analysis tool, was used to predict the GO, which reveals essential component of the gene via high-throughput investigation. They are (i) biological process (BP), (ii) molecular function (MF), and (iii) cellular component (CC) of the gene function to find the pathways of DEGs using KEGG. KEGG is a popular database with a plethora of information on genomes, biological pathways, drugs, and chemical substances.

### 2.3. PPI and Module Analysis

A PPI network was constructed to identify the depth of closeness between genes via the STRING database with a high certainty score of 0.700 as the cutoff condition [9]. Assembling of a PPI network was coordinated for the recovery of interfacing qualities. The default settings were used for all other parameters. Outcome of the hub genes were notified with the degree of every single gene. The retrieved PPI network was converted in gto.tsv file format. The .tsv file was uploaded into the plug-in CytoHubba, which is a component in version 3.8.2 of the Cytoscape software [10]. Hub genes were identified based on the highest degree score from the protein-protein interaction result. The plug-in MCODE (molecular complex detection) in Cytoscape is used to identify the clustering nodules of hub genes [11]. Hub genes were defined with at least 10 gene degrees in the PPI network, and all those network diagrams of key genes were visualized.

### 2.4. Validation of Hub Genes

GEPIA2 was used to detect the expression level in the middle of tumor vs. normal in gastric cancer samples [12]. Based on the node rank and position, top 10 genes were selected and entered into the GEPIA2 tool to confirm the expression in TCGA-STAD (The Cancer Genome Atlas-Stomach Adenocarcinoma). Interactions between the hub genes were visualized using a box plot.

### 2.5. Survival Analysis

The Kaplan–Meier plotter was used to evaluate the impact in 54,675 genes on endurance utilizing malignant growth test (10,461), including Bosom cancer (5143), ovarian cancer (1816), pulmonary cancer (2437), gastric cancer (1065) [13]. According to these overall survival details, the genes were sorted from high to low expression based on the TCGA database. The *P* value log rank was determined and shown in the site page with 95% confidence interval in HR (hazard ratio).

## 3. Results

### 3.1. DEGs in Gastric Cancer

This research includes both tumor tissue (TT) and normal tissue (NT). Totally, 56 samples (tumor 28 and normal 28) in GSE161533 and 132 samples (tumor 111 and normal 21) in GSE54129 were involved in DEG (differentially expressed gene) analysis (Table 1). DEGs expression profiles were notified and showed in a volcano plot (Figure 2) with heat map outcome (Figure 3). Likewise, Venn analysis (genevenn.sourceforge.net) was utilized to retrieve the interacting genes in DEGs profile (Figure 4). At last, overall, 173 genes were identified to be differentially expressed, with 112 upregulated genes and 61 downregulated genes (Table 2).

### 3.2. Analysis of Gene Ontology and KEGG Pathway

The analysis of GO revealed that DEGs were mostly in association with positive regulation by a host of viral process (GO: 0044794), positive regulation of granulocyte differentiation (GO: 0030854), negative regulation of histone H_3_–K_9_ methylation (GO: 0051573), modulation of host of viral process (GO: 0044788), and biotin metabolic process (GO: 0006768) (Figure 5(a)). Molecular function revealed that DEGs altogether improved G-quadruplex DNA binding (GO: 0051880), DNA-(apyrimidinic (or) apurinic site) endonuclease activity (GO: 0003906), 3′-5′ exodeoxyribonuclease activity (GO: 0008296), D-loop DNA binding (GO: 0062037) and ketosteroid monooxygenase activity (GO: 0047086) (Figure 5(b)). DEGs, U4 snRNA (GO: 0005687), alveolar lamellar body (GO: 0097208), multivesicular body lumen (GO: 0097486), U7 snRNP (GO: 0005683), and MLL1 complex (GO: 0071339) enhanced in the cellular component (Figure 5(c)). Most of the DEGs are fundamentally enhanced in cell cycle regulation, cell proliferation, and binding and transcriptional activity, and significantly enhanced in nucleotide excision repair, homologous recombination, DNA replication, complement and coagulation cascades, and base excision repair (Figure 5(d)).

### 3.3. Hub Genes Identification

In the PPI network, a sum of 107 nodes, 47 edges, 0.879 avg. node degree, and 0.332 avg. local clustering coefficient, and 0.0903 PPI enrichment *p* value were emerged (Figure 6) [14]. According to the STRING database's reference value (PPI enrichment *p* value = 1.0e-16), the created PPI network in this study contains much more acceptable interactions. The top ten hub genes were validated by the interaction score of CytoHubba (Figure 7). Following are the CytoHubba outcomes of hub genes in gastric cancer: DNA polymerase epsilon, catalytic subunit (POLE), mitotic checkpoint serine/threonine-protein kinase BUB1 beta (BUB1B), DNA polymerase delta subunit 4 (POLD4), complement 3 (C3), Bloom, Syndrome, RecQ helicase-like (BLM), chaperon containing TCP1 subunit 7 (eta) (CCT7), pre-mRNA processing factor 31 (PRPF31), APEX nuclease (multifunctional DNA enzyme repair 1), proteasome (prosome, macropain) subunit alpha type 7 (PSMA7), and cell division control protein 45 homolog (CDC45).

### 3.4. Overall Survival Analysis

Survival analysis was performed utilizing the KM plotter to endorse the prognostic biomarkers of the ten putative hub genes. On the KM plotter, a total of 876 GC patients were available for overall survival. High mRNA articulation levels (Table 3) were substantially linked with overall survival rate, as shown in (Figure 8). Findings confirmed with prognostic value of 10 hub genes as well as the links between genes in gastric cancer metastasis. The survival curves showed the significant DEGs, including POLE, POLD4, C3, BLM, and PRPF31, which were identified. The identification displayed that to be related with unfavorable survival rates in gastric cancer. Then, the GEPIA database was utilized (Figure 9), and the top ten genes in the STAD samples in the TCGA database by degree value BUB1B, CCT7, APEX1, PSMA7, and CDC45 were found to be strongly expressed.

## 4. Discussion

Totally, 173 DEGs were separated into 3 categories based on functional annotation in gene ontology: (i) BP, (ii) MF, and (iii) CC. The consequences of useful analysis of enrichment demonstrate that critical DEGs in gastric carcinoma patients were engaged with gene ontology, biological process such as positive regulation by a host of viral process and granulocyte differentiation, negative regulation of histone H_3_–K_9_ methylation, modulation of host of viral process, and biotin metabolic process. From this analysis, 112 upregulated and 61 downregulated DEGs in gastric malignancy is separated from two GEO datasets.

Overexpression of BUB1B, CCT7, APEX1, PSMA7, and CDC45 was revealed and showed great prognostic variables in gastric cancer. The POL DNA polymerase enzyme complex synthesizes the leading strand, and the key catalytic and proof reader component of the complex was encoded by POLE [15]. The proofreading mechanism detects and replaces incorrect bases in the daughter strand as a result of unsuccessful complementary mating with the parental strand. POLE's high-fidelity base incorporation, paired with exonuclease proofreading activity, results in low mutation rate [16]. The part of BUB1B, (encoding BUBR1) malignancy cells is as yet questionable as a designated spot for fitting chromosomal isolation and forestalling detachment of copied chromosome in typical cells. BUB1B in human adenocarcinoma [17] and lung cancer which indicates worse survival rate and metastasis [18]. Overexpression of BUB1B has been linked to the movement and recurrence of gastric tumor [19] including glioblastoma, ductal adenocarcinoma, prostate disease, gastric adenocarcinoma, and hepatocellular carcinoma [31] as well as many other cancers [30]. The complement system (C3) is involved in progression of malignancies along with bladder, hepatocellular, and cervical carcinomas. This paper is the first discloser of the prevalence of supplement depletion in GC, in addition to its predictive importance for quick and long-term effects [28]. The BLM gene makes the Bloom syndrome, RecQ helicase-like helicase protein, which would be needed for replication of DNA and genomic respectability conservation. The RecQ helicase family has developed over the long run, and 3′ to 5′ DNA helicase in BLM that has a place with it.

Therefore, cells inadequate in BLM had a ten times expansion in chromatid breakage, sister chromatid hybrid development, and mitotic recombination [20]. PRPF31 (pre-mRNA processing factor 31) is an important protein required for pre-mRNA splicing between 4/U6 disnRNA and the U5 snRNP [21]. PRPF31 has been found to have loss of function, leading in lower quantities of active snRNPs and worse splicing efficiency [22]. APEX1 (APEX nuclease (multifunctional DNA repair enzyme) 1) may assume a part in malignancy by repairing DNA harm [23]. As a result, genetic abnormalities affecting APEX1's ability to repair itself are frequently considered reasonable candidates for functional research. The transition between 1349th base pair *T* allele and 5th exon of the APEX1 gene and *G* allele has been widely analyzed in conjunction with a variety of cancers, including pulmonary cancer, bosom caner, and bladder cancer (ASP 148Glu, rs1130409), resulting in the replacement of 148th amino acid aspartate (Asp) to glutamate (Glu) (Asp 148Glu, rs1130409) [33]. Multiple forms of tumors have been shown to have the 20q region amplified [24, 34]. The component of the 20S proteasome core complex, which is involved in eukaryotic cell degrade proteins via the ubiquitin-proteasome pathway. The protein complex, which has a molecular mass of 2,000 kDa, is made up of a 20S proteolytic core and one or two 19S regulatory complexes [25, 32]. To form a replication commencement complex, numerous proteins must be assembled and meticulously coordinated into the start of replication. The human CDC45 protein (hCdc45) is needed for both the establishment and portability of the replication fork [26]. CDC45 is required during the DNA replication cycle, according to numerous studies, and CDC45 overexpression has been linked to malignancy cell proliferation [27].

## 5. Conclusion

We identified certain critical genes and described the biological process and signaling pathway that are nearly associated with gastric cancer formation and progression systematically. These genes had not yet been discovered recently, although they could be crucial in gastric cancer. Outstandingly, contrasted with all other worldwide examination, dissecting prognostic results on BUB1B, CCT7, APEX1, PSMA7, and CDC45 separately in our study yielded conflicting ends. Overall, results proved that example sizes were inconsistent. Furthermore, thorough investigation on BUB1B, CCT7, APEX1, PSMA7, and CDC45 is justified. From this analysis, the top ten hub genes are upregulated genes. Therefore, this reduces the survival of gastric cancer patients, and also it can improve the survival rate and reduce the death rate which concentrate on suppressing or controlling this gene's function.

## Figures and Tables

**Figure 1:** Workflow for identification of strong prognostic biomarker genes in mGC.

**Figure 2:** DEGs between GC samples and normal samples: volcano plot. (a) GSE54129 and (b) GSE161533 show the expressions of the upregulatory genes which are shown in red colour, the downregulatory genes are shown in blue colour, and nonsignificant genes are shown in grey colour.

**Figure 3:** The differentially expressed genes (DEGs) are displayed in a heat map. (a) GSE54129 and (b) GSE161533 are shown with hierarchical grouping. High expression level is expressed in red colour and low expression level is addressed in blue colour.

**Figure 4:** The overlapping between two GEO datasets is shown by a Venn diagram. The Venn diagram indicates the overlaps in the (a) upregulatory genes and (b) downregulatory genes.

**Figure 5:** Pathway enrichment results: GO term and KEGG pathway enhancement examinations performed utilizing Enrichr. The best 10 enriched in the biological process, molecular function, cellular component, and KEGG pathway for DEGs. The *x*-axis addresses the number of genes and the *y*-axis addresses the (a) BP, (b) MF, (c) CC, and (d) KEGG pathway in names.

**Figure 6:** STRING protein-protein interaction network. The network contains 107 nodes and 47 edges, with 0.700 confidence score, 0.879 avg. node degree, 0.332 avg. local clustering coefficient, and PPI enrichment *p* value = 0.0903. The pearl shape indicates the genes, the lines showed the interaction of protein between the genes, inside the circle is protein, and the colour of the line represents the proof of interaction between the proteins.

**Figure 7:** Cytoscape software used to retrieve the top hub genes. Node colour gives an idea for connection of degree. The major ten hub gene shows the colour change from red to yellow. The red colour shows the highest degree, light orange shows the intermediate one, and lowest degree reflects the yellow colour. Rank node is shown from the top hub genes.

**Figure 8:** Expression of the hub genes in the TCGA database. The box plots indicate the expression level of the gene (mGC) (A–J) POLE, BUB1B, POLD4, C3, BLM, CCT7, PRPF31, APEX1, PSMA7, and CDC45 in GEPIA. The red colour represents in tumor and grey colour represent in normal.

**Figure 9:** Overall survival analysis of the key genes in GC patients drawn by KM plotter. The gene expression of the patients was classified into groups based on the two medians: high-expression median and low-expression median. The genes were (A–J) POLE, BUB1B, POLD4, C3, BLM, CCT7, PRPF31, APEX1, PSMA7, and CDC45 mRNA expression. Kaplan–Meier survival plots show the higher expression of up regulatory genes (BUB1B, CCT7, APEX1, PSMA7, and CDC45). The survival curve of the other five up regulatory genes (POLE, POLD4, C3, BLM, and PRPF31) shows the lower expression in GC patients.

**Table 1:** Details of GEO gastric cancer data.

	Details of GEO gastric cancer data			
Dataset ID	Platform	Tumor	Normal	Update date
GSE161533	GPL 570 [HG-U133_Plus_2] Affymetrix human genome U133 plus 2.0 array	28	28	Nov 19, 2020
GSE54129	GPL 570 [HG-U133_Plus_2] Affymetrix human genome U133 plus 2.0 array	111	21	Mar 25, 2019

**Table 2:** Screening DEGs in gastric cancer.

DEGs	Gene terms
Upregulatory	ABCF1, ACIN1, ACTRT3, AKR1C3, ALOX12P2, ANXA5, APEX1, APOL1, AXIN1, BAMBI, BLM, BUB1B, C17orf100, C3, CCRL2, CCT7, CDC123, CDC37, CDC45, CEMIP, CHCHD5, CKAP2L, CKS2, CNN2, COLGALT1, CPSF6, CRIP2, CSE1L, CTSH, CWC15, DEXI, DNLZ, DNMT1, DPF2, DRAP1, DSCR9, E2F6, ENO2,FAM168 A, FBXL15, FCHSD1, F1BP, FLYWCH2, FOSL1, GEM, GZMH, HAUS8, HAX1, HCLS1, HTRA2, IGF2R, IL2RA, IMPDH1, JUNB, KDM1A, KIAA0930, KIF2A, KRT23, LDHA, LOC101927330, LOC648987, LONP1, LRRC15, MAMSTR, MBTPS1, MLLT11, MNAT1, MRPL52, MVB12 A, NAA40, NBL1, NDUFA3, NFIL3, NOC2L, NTHL1, PC, PCDHB2, PGBD5, PIGH, PLA2G2A, PLAU, PLIN2, POLD4, POLE, PPIB, PRPF31, PSMA7, PUM1, RALGDDS, RIPK2, SELPLG, SERPING1, SHCBP1, SLC5A6, SNRPF, STOM, SURF2, TLR1, TP53I11, TRIM28, UBE2L6,USP1, USP11, VEGFC,WDR54,YTHDF3, AS1,ZMYND19,ZNF200,ZNF511, ZNF783, ZYG11 A

Downregulatory	ABT1, AK6, ALDOC, ALOX12, ARHGAP5-AS1, ARL4A,BLOC1S4, C4orf33, CCDC85 C, CDA, CDK20, CGGBP1, CIPC, CRNDE, CRNKL1, DENND6A, DHRS7B, DSCR4, DUSP22, ECHS1, ETV3, FAAH2, FAM117 A, IRAK4, ITGAD, KHDC1, KIF12, LINC00685, LOC93622, MBD5, MIEF2, MYL5, NRIP2, OTUD3, P2RX1, PARP4, PIK3C2G, PNP, PRSS16, RNF186, SERTAD4-AS1, SLC16A9, SMIM24, SP5, SPATA32, SRGAP2C, STAP2

**Table 3:** Overall survival analysis of the top 10 upregulatory genes of GC patients in GSE161533 and GSE54129.

Gene	HR^*∗*^ (95% CI^*∗∗*^)	*P* value
POLE	1.66 (1.4–1.98)	9.7e-09
BUB1B	0.75 (0.62–0.92)	0.0059
POLD4	1.46 (1.23–1.73)	1.2e-0.5
C3	1.23 (1.03–1.48)	0.024
BLM	1.22 (1.01–1.48)	0.038
CCT7	0.66 (0.55–0.79)	5.2e-0.6
PRPF31	1.36 (1.15–1.62)	0.00041
APEX1	0.88 (0.74–1.06)	0.19
PSMA7	0.61 (0.52–0.72)	9.6e-09
CDC45	0.78 (0.66–0.93)	0.0047

^*∗*^HR, hazard ratio; ^*∗∗*^CI, confidence interval.

## Data Availability

Sufficient data have been included in the manuscript. Additional data can be kindly requested from the corresponding author.

## Abbreviation

APEX1: APEX nuclease (multifunctional DNA repair enzyme) 1
BP: Biological process
BUB1B: Mitotic checkpoint serine/threonine-protein kinase BUB1 beta
CC: Cellular component
CDC45: Cell division control protein 45 homolog
CCT7: Chaperon containing TCP1 subunit 7
DEG: Differentially expressed gene
GC: Gastric cancer
GEO: Gene expression omnibus
GEPIA: Gene Expression Profiling Interactive Analysis
GO: Gene ontology
KEGG: Kyoto Encyclopedia of Genes and Genomes
KM plotter: Kaplan–Meier plotter
MF: Molecular function
NT: Normal tissue
PPI: Protein-protein interaction
PSMA7: Proteasome (prosome, macropain) subunit alpha type 7
STRING: Search Tool for the Retrieval of Interacting Genes
STAD: Stomach adenocarcinoma
TCGA: The Cancer Genome Atlas
TT: Tumor tissue.
